# Decreased Spp1 Expression in Acute Myocardial Infarction after Ischemia and Reperfusion Injury

**DOI:** 10.1155/2021/3925136

**Published:** 2021-08-13

**Authors:** Ling Li, Jungang Huang, Zongkai Zhao, Zhuzhi Wen, Kang Li, Tianjiao Ma, Lisui Zhang, Junmeng Zheng, Shi Liang

**Affiliations:** Department of Cardiovascular Surgery, Sun Yat-sen Memorial Hospital, Sun Yat-sen University, Guangzhou 510120, China

## Abstract

**Background:**

With the progress of shock therapy and the establishment and promotion of methods such as thrombolytic therapy and percutaneous coronary intervention (PCI), many tissues and organs have been reperfused after ischemia which may cause even worse disorder called ischemia-reperfusion injury (IRI). mRNAs have been found to have significant impacts on ischemia-reperfusion through various mechanisms. In view of the accessibility of mRNAs from blood, we aimed to find the association between mRNA and ischemia-reperfusion.

**Methods:**

We used the GSE83472 dataset from the Gene Expression Omnibus (GEO) database to find differential RNA expression between ischemia-reperfusion tissue and control samples. In addition, Gene Ontology (GO) annotation and Kyoto Encyclopedia of Genes and Genomes (KEGG) pathway analyses were performed to find the biological property of 449 RNAs from GSE83472 via the Database for Annotation, Visualization, and Integrated Discovery (DAVID). Besides, Gene Set Enrichment Analysis (GSEA), a tool to find the pathway orientation of a gene set, was used for further study in the four most significant KEGG pathways. Furthermore, we constructed a protein-protein interaction (PPI) network. In the end, we used quantitative reverse transcription-polymerase chain reaction (qRT-PCR) and western blotting to measure and compare the expression of Spp1 in patients who accepted percutaneous coronary intervention.

**Results:**

The bioinformatics analyses suggested that Spp1 was a hub gene in reperfusion after ischemia. The qRT-PCR result showed that the Spp1 expression was significantly downregulated in ischemia-reperfusion cells after PCI compared with normal samples and so as the western blotting.

**Conclusion:**

Spp1 might play an essential role in acute myocardial infarction after ischemia and reperfusion injury.

## 1. Introduction

Myocardial infarction (MI) ranks first among the heart vascular events around the world; the timely and effective recovery of coronary artery blood flow is an effective method for the treatment of ischemic heart disease [1]. However, the process of blood reperfusion may cause myocardial tissue structure, energy metabolism, electrophysiology, and heart function damage; this phenomenon is called myocardial ischemia-reperfusion [2]. The underlying mechanism is various. The accumulation of lactate, protons, and NAD+ in ischemic tissue causes the decrease of pH. The H+ ions were extruded in exchange for Na+ through the Na^+^/H^+^ exchanger. Consequently, the cell extrudes Na^+^ in exchange for Ca^2+^ by the Na^+^/Ca^2+^ exchanger. The surplus Ca^2+^, flowing into the mitochondria, may activate the Ca^2+^/calmodulin-dependent protein kinases pathologically [3]. A recent study considered that the IRI promoted the production of proinflammatory cytokines and induced proapoptotic pathways of the unfolded protein response (UPR) [4]. Secreted phosphoprotein‐1 (Spp1), also called as osteopontin (OPN), is a protein secreted by the SPPL gene encoded on human chromosome 4q22.1 which interacts with a number of adhesion receptor-binding motifs including a C-terminal CD44v6 domain and thrombin-cleaved N-terminal integrin domain [5]. Recent studies show that Spp1 is an extracellular matrix protein closely related to tumors, which is expressed at a high level in many tumors and involved in the regulation of tumor invasion, metastasis, apoptosis inhibition, and angiogenesis [6]. In our study, differentially expressed RNAs (DE-RNAs) were identified from the GSE83472 dataset, and we found Spp1 as the candidate associated with IRI. Then, we analyzed the functional enrichment of specific biologic processes via DAVID. A PPI network was generated and measured for finding the hub gene associated with IRI. Finally, we validated the downregulation of Spp1 expression in ischemia-reperfusion patients after PCI.

## 2. Methods

### 2.1. Data Download and Clinical Samples

We obtained the GSE83472 dataset from GEO (http://www.ncbi.nlm.nih.gov/geo/) [7]. The GSE83472 dataset, including 8 mouse SHAM (4 WT and 4 AKIP_TG) and 8 mouse IR (4 WT and 4 AKIP1_TG) where ischemia/reperfusion injured, was used to identify differential gene expression for mice with I/R injury. Meanwhile, we gathered clinical samples from 9 males and 7 females, with an average age of 53.6 ± 8.4 years, who accepted percutaneous coronary intervention because of acute myocardial infarction from 2018 to 2020. The whole blood samples from patients and healthy people were gathered. The guidelines of the Ethics Committee of Sun Yat-sen University, Sun Yat-sen Memorial Hospital (SYSEC-KY-KS-2021-070), were obeyed.

### 2.2. Data Processing

We used the R language and applied the R package of “limma” to process the GSE83472 RAW dataset (*p* < 0.05). Then, we screened out DE-RNAs according to the criteria gene expression values. Furthermore, we made volcano plot and heat map for differential expression genes and the analysis results.

### 2.3. GO Functional Annotation and KEGG Pathway Enrichment Analysis

To analyze GO terms of DE-RNAs and the enrichment in KEGG pathways, we used DAVID to reveal potential functions and the biological property of DE-RNAs with *p* < 0.05 [8].

### 2.4. GESA

For further study, GESA, a tool for learning the enrichment in specific functional gene sets, was performed using the online tool available at http://software.broadinstitute.org/gsea. The gene sets of C2 (curated) KEGG, C5 (GO) cellular components, C5 (GO) biological processes, and C5 (GO) molecular functions were used to find the function of DE-RNAs through the R package cluster Profiler [9].

### 2.5. PPI Network Construction

To explore the association of DE-RNAs, we subsequently generated the PPI biological network and evaluated the interaction through the STRING database (https://string-db.org/). In addition, Cytoscape software was used for the visualization of interactions and finding the hub gene in functional networks [10]. Finally, the hub genes were verified by the MCODE method, and the CytoHubba application was used to rank the gene and construct a network by its score [11].

### 2.6. qRT-PCR Analysis

We synthesized cDNA by reverse-transcribing RNA by using RNA Transcription Kit (Western Biotech, Chongqing, China). The forward primers and reverse primers are listed in Table 1. Then, we used SYBR Green Mix (Yeasen Biotech Co., Ltd.) to perform qRT-PCR on a Roche Real-Time PCR System according to the manufacturer's instructions. We calculated fold changes in RNA expression using the 2^−ΔCt^ (2^−[(Ct of gene)−(Ct of U6)]^) method as previously described [12].

### 2.7. Western Blotting Assay

Cells were collected and resolved on ice with RIPA buffer. After that, the protein samples were separated in 10% polyacrylamide SDS-PAGE and transferred onto a polyvinylidene fluoride (PVDF) membrane [13]. After transferring, we blocked the PVDF membranes with 5% bovine serum albumin (BSA). We used osteopontin (Abcam, ab166709) and GAPDH (Cell Signaling Technology) as primary antibodies to incubate blocked membranes at 4°C overnight and horseradish peroxidase as the secondary antibody at room temperature. Finally, samples were detected by using the ECL detection kit (Yeasen Biotech Co., Ltd.) [14].

### 2.8. Statistical Analysis

For the qRT-PCR in clinical samples, Student's *t*-test was performed using GraphPad 7.0. We used R software (https://www.r-project.org/) to perform bioinformatics analysis. The values were shown as mean ± standard deviation and then analyzed using two-tailed Student's *t*-tests. A *p* value of <0.05 was considered to indicate a statistically significant difference.

## 3. Results

### 3.1. Bioinformation Analysis from the GSE83472 Dataset

We screened out DE-RNAs according to the criteria that |Log2FC| > 1, where FC represented fold change, and *p* value <0.05. Subsequently, 221 upregulated DE-RNAs and 318 downregulated DE-RNAs were identified. The result was shown in the volcano plot and heat map, respectively (Figures 1(a) and 1(b)). To identify the function of target genes, we utilized DAVID to perform GO annotation and KEGG pathway analyses. The top 4 significant GO terms and KEGG pathways are shown in Figures 1(c)–1(f). The significantly enriched entries for the biological process were the negative regulation of the apoptotic process (Figures 1(c)–1(f)). The most enriched cellular component was functions in the cytoplasm (Figure 1(d)), and protein binding was dominant in the molecular function (Figure 1(e)).

### 3.2. Enrichment Analysis by GSEA

GSEA was performed to evaluate the GO gene sets and KEGG signaling pathway gene sets between IR and NIR. Twenty signaling pathways were differentially enriched, among which the largest enrichment score (ES) was propanoate metabolism, valine, leucine, and isoleucine degradation, Parkinson's disease, citrate cycle (TCA cycle), mitochondrial respiratory chain complex 1 biogenesis, mitochondrial respiratory chain complex assembly, fatty acid beta oxidation using acyl-CoA dehydrogenase, mitochondrial ATP synthesis coupled proton transport, NADH dehydrogenase complex, proton-transporting ATP synthase complex, respiratory chain, inner mitochondrial membrane protein complex, oxidoreductase activity acting on NADPH quinone or similar compound as the acceptor, acyl-CoA dehydrogenase activity, NAD-ADP ribosyl transferase activity, and oxidoreductase activity acting on NADPH (Figures 2(a) and 2(c)–2(e)), and the largest negative enrichment score (NES) was ribosome, NOD-like receptor signaling pathway, DNA sensing pathway, and pathogenic *Escherichia coli* infection (Figure 2(b)).

### 3.3. Spp1 Was Identified as the Hub Gene Associated with Ischemia, Cell Injury, and Inflammation

A PPI network including 400 nodes and 2085 edges with association confidence score >0.4 was constructed to distinguish the connection among 539 DE-RNAs by the STRING database. Within the 26 genes identified by the MCODE application, the Spp1 gene had a high score (Figure 3(a)). As shown in the figure, the hub gene network and functional clustering indicated Spp1 as the hub gene associated with IRI (Figures 3(b) and 3(c)).

### 3.4. Spp1 Was Downregulated in Ischemia-Reperfusion Samples after PCI

We quantified the expression levels of Spp1 by qRT-PCR in the whole blood cells (Figure 4(a)). The expression of Spp1 in ischemia-reperfusion samples after PCI was significantly decreased compared to the control. The western blotting result indicated the downregulation of Spp1 expression in ischemia-reperfusion samples at the protein level (Figure 4(b)).

## 4. Discussion

Tissue lesion caused by ischemia is the main cause of fatal diseases, such as MI and stroke [15]. MI can lead to the gradual development of heart failure, chronic ischemic heart disease, the result of persistent or repeated aggravation of myocardial ischemia, and hypoxia caused by severe coronary artery atherosclerotic stenosis [16]. In gross appearance, the thickness of the heart wall may be normal, with multifocal white fibrous bands or transmural scars. The endocardium thickens and loses its normal luster and sometimes with mural thrombus. In addition, MI can induce multifocal myocardial fibrosis and myocardial fiber hypertrophy. During the rescue and treatment of ischemic diseases, scientists gradually discovered that the main lesion to tissues is not the ischemia itself, but after the blood supply is restored, excessive free radicals attack this part of the tissue. This phenomenon is called ischemia/reperfusion injury [17].

Spp1, known as osteopontin, is an extracellular matrix protein [18]. There are few previous studies on the relationship between Spp1 and IRI. A recent study has shown that inhibition of Spp1 expression can inhibit cell proliferation, which is a potential target for cancer therapy. Besides, scientists indicated that the postnatal inhibition of Spp1 can reduce fibrosis and facilitate motor function in DMD (Duchenne muscular dystrophy) mice through promoting TGF-*β* [19]. Also, the decrease of Spp1 expression induced by ischemia can damage neovascularization, while the overexpression of Spp1 can increase angiogenesis [20]. Furthermore, as a key mediator of neovascularization after ischemia, Spp1 would be a new target for inducing angiogenesis. The ability to form new collateral circulation is closely related to reducing long-term cardiac mortality in patients with AMI and stable CAD [21]. These studies provide clues for us to explore the relationship between Spp1 and IRI.

In this study, we downloaded the GSE83472 database for differential analysis. Afterwards, 539 RNAs were identified as DE-RNAs and used to construct the PPI network through the STRING database. A network of 400 nodes and 2085 edges was obtained for further study. According to the GO/KEEG analyses and GSEA, it was indicated that these proteins were mostly located in the cytoplasm and involved in the negative regulation of the apoptotic process and transportation. Furthermore, we identified 26 hub genes by the MCODE application of Cytoscape where the Spp1 gene achieved a high score. Besides, the hub gene network and functional clustering suggested a strong connection between Spp1 and IRI. In the end, we verified our finding in the clinical samples. Both western blotting and qRT-PCR analyses revealed the downregulation of Spp1 in acute myocardial infarction samples after IRI which may suggest the negative correlation between Spp1 and IRI. Overall, we considered that Spp1 might be regarded as a potential diagnostic biomarker in IRI because of the availability in serum and it can avoid several invasive tests.

There remain several limitations to our study such as the possible bias when analyzing DE-RNAs due to the small size of the dataset. Similarly, more blood samples from different centers can help us get more accurate results of *in vitro* experiments. Another limitation is the animal model; we did not establish a suitable animal model to validate the Spp1 level *in vivo*. Also, the related signaling pathway was needed to detect for revealing the molecular mechanism. In brief, the study on the regulation and potential pathway of genes is not complicated enough. If conditions permit, we will focus on the regulation of downstream target genes and the potential signaling pathway of Spp1.

## 5. Conclusions

Our study aimed to clarify the association of Spp1 with IRI through the bioinformatics analysis of the GEO database, GO/KEEG analyses, and GSEA. Furthermore, we figured out that the expression of Spp1 was downregulated in *in vitro* experiments by qRT-PCR and western blotting analyses. In the rat model of myocardial IRI, bioinformatics and integration of gene expression profiles indicated Spp1 as a hub gene closely associated with myocardial IRI, supporting the potential role in myocardial IRI.

## Figures and Tables

**Figure 1:** Bioinformation analysis from the GSE83472 dataset. (a) Volcano plot of DE-RNAs from the GSE83472 dataset. Red dot represented upregulated RNAs, and yellow dot represented downregulated RNAs. (b) Heat map of hierarchical clustering analysis for DE-RNA expression. Red represented greater expression, and blue represented less expression. (c–f) The top 15 significant KEGG pathways and GO terms related to the biological process, cellular component, molecular function.

**Figure 2:** Enrichment analysis by GSEA. (a) In gene sets of KEGG, GSEA revealed that the genes of IR were mainly enriched in propanoate metabolism, valine, leucine, and isoleucine degradation, Parkinson's disease, and citrate cycle (TCA cycle). (b) In gene sets of KEGG, GSEA revealed that the genes of IR were mainly negatively enriched in ribosome, NOD-like receptor signaling pathway, DNA sensing pathway, and pathogenic *Escherichia coli* infection. (c–e) In gene sets of GO, GSEA revealed that the genes of IR were mainly enriched in mitochondrial respiratory chain complex 1 biogenesis, mitochondrial respiratory chain complex assembly, fatty acid beta oxidation using acyl-CoA dehydrogenase, mitochondrial ATP synthesis coupled proton transport, NADH dehydrogenase complex, proton-transporting ATP synthase complex, respiratory chain, inner mitochondrial membrane protein complex, oxidoreductase activity acting on NADPH quinone or similar compound as the acceptor, acyl-CoA dehydrogenase activity, NAD-ADP ribosyl transferase activity, and oxidoreductase activity acting on NADPH. (a) GSEA (KEGG). (b) GSEA (KEGG). (c) GSEA (biological process). (d) GSEA (cellular component). (e) GSEA (molecular function).

**Figure 3:** Spp1 was identified as the hub gene associated with ischemia, cell injury, and inflammation. (a) The PPI network indicated the interaction of 27 hub genes. (b) Hub gene network was obtained through Cytoscape, and Spp1 obtained a high score. (c) The functional clustering indicated Spp1 as a hub gene involved in ischemia, cell injury, and inflammation in the connection tissue using the Metascape database.

**Figure 4:** Downregulation of Spp1 expression in ischemia/reperfusion after PCI. (a) qRT-PCR analysis showing the expression of Spp1 in ischemia-reperfusion samples after PCI (square shape) compared to normal samples (circle shape). ^*∗*^*p* < 0.05. (b) Western blot indicating that Spp1 protein levels were significantly downregulated in ischemia-reperfusion cells after PCI compared with normal cells.

**Table 1:** Primers.

SPP1	Forward	CTCCATTGACTCGAACGACTC
	Reverse	CAGGTCTGCGAAACTTCTTAGAT
GAPDH	Forward	ACAACTTTGGTATCGTGGAAGG
	Reverse	GCCATCACGCCACAGTTTC

## Data Availability

All the datasets used to support the findings of this study are available from the corresponding authors upon request.
